# Clinical Efficacy of Ulinastatin Combined with Meglumine Adenosine Cyclophosphate in the Treatment of Acute Myocardial Infarction

**DOI:** 10.1155/2022/2172412

**Published:** 2022-04-18

**Authors:** Zhenying Zhang, Xiaojing Sun, Jiagui Ma, Qiaoyan Ma, Qian Cao, Liu Zhang, Lizhong Wang

**Affiliations:** Cardiac Rehabilitation Center, Beijing Rehabilitation Hospital, Capital Medical University, Beijing 100144, China

## Abstract

Ulinastatin, a common adjuvant drug in the clinical treatment of acute circulatory failure, has a good effect on various inflammatory diseases. In this study, we aim to explore the clinical efficacy of ulinastatin combined with meglumine adenosine cyclophosphate in patients with acute myocardial infarction (AMI) and its effect on cardiac function and endothelial function of patients. 100 AMI patients treated in our hospital (February 2020-October 2020) were randomly chosen and divided into group J and group Q, with 50 cases in each group. Group Q was treated with meglumine adenosine cyclophosphate only, while group J was treated with ulinastatin combined with meglumine adenosine cyclophosphate to compare the treatment efficiency, cardiac structure indexes, cardiac systolic function, blood lipid levels, vascular endothelial function, QLI (quality of life) scores, BI indexes, and FMA (motor function) scores between the two groups. The treatment efficiency, QLI score, BI index, and FMA score in group J were notably higher compared with group Q (*P* < 0.05). The cardiac structure indexes, cardiac systolic function, blood lipid level, and vascular endothelial function in group J were notably better compared with group Q (*P* < 0.05). Ulinastatin combined with meglumine adenosine cyclophosphate can obviously enhance the therapeutic effect of AMI patients and improve the endothelial function and cardiac function of patients, which is very promising in this medical area.

## 1. Introduction

Ulinastatin is a common adjuvant drug, which acts as a protease inhibitor to treat acute circulatory failure and other diseases. And ulinastatin is a common drug used in clinical treatment of acute pancreatitis and other diseases, which also plays a key role in the treatment of tumor patients and the auxiliary rescue of acute debilitating diseases. The application of ulinastatin can protect the kidney of patients needing chemotherapy being affected by chemotherapy as much as possible, thus improving the therapeutic effect [1–3]. Meglumine adenosine cyclophosphate is a cardiotonic drug specially to treat acute heart diseases, which is widely used in acute heart failure, acute myocardial infarction, myocarditis, and other diseases. And it is also a drug specially used for the treatment of heart diseases such as coronary heart disease, myocardial infarction, heart failure, and angina pectoris, with wide application in clinic due to its significant clinical effect and less side effect. Cardiac structure indexes included aortic diameter (AD), posterior wall thickness during systole (PWTs), interventricular septal thickness (IVS), and left ventricular internal diameter at end-systole (LVIDs) [4–6].

At present, meglumine adenosine cyclophosphate is mainly applied in clinic by intravenous drip after dilution with glucose injection. Acute myocardial infarction (AMI) is a common acute heart disease in middle-aged and elderly people with rapid onset, fast development, and high mortality. If patients are diagnosed with AMI, anticoagulant and antithrombotic measures will be taken immediately, and surgical treatment will be provided if necessary. Moreover, middle-aged and elderly people are prone to AMI because their heart function declines with age [7–9]. After the onset, patients should go to the hospital for medical treatment immediately, so as to shorten the time from onset to treatment as much as possible. Shorter time indicates less impact of the disease on patients and smaller treatment risk [10–12]. It has been reported that the combination of ulinastatin and meglumine adenosine cyclophosphate in AMI patients can significantly enhance the therapeutic effect [13–15]. Song et al. [16] proposed a study in which AMI patients were divided into group A treated with meglumine adenosine cyclophosphate and group B treated with ulinastatin combined with meglumine adenosine cyclophosphate. Therefore, weakened cardiac systolic function will seriously affect the blood circulation and even cause death in patients [17, 18].

Therefore, we aim to investigate the application effect of ulinastatin combined with meglumine adenosine cyclophosphate in the treatment of AMI patients and its effect on cardiac function and endothelial function. And AMI patients were treated with meglumine adenosine cyclophosphate only and meglumine adenosine cyclophosphate combined with ulinastatin, reported as below. And we compare the treatment efficiency, cardiac structure indexes, cardiac systolic function, blood lipid levels, vascular endothelial function, QLI scores, BI indexes, and FMA scores in our study.

## 2. Materials and Methods

### 2.1. General Information

One hundred AMI patients treated in our hospital (February 2020-October 2020) were randomly chosen and divided into group J and group Q, with 50 cases in each group. The patients were aged 55-73 years old in group J and 56-74 years old in group Q. No statistical significance in gender, age, medical history, and other general data was found between the two groups (*P* > 0.05, Table 1).

### 2.2. Inclusion/Exclusion Criteria

#### 2.2.1. Inclusion Criteria

1. The patients met the clinical manifestations of AMI
2. The patients were aged no less than 18 years old
3. The patients had no history of drug allergy and drug abuse and no bad habits
4. The patients had no severe cardiovascular and cerebrovascular diseases recently
5. This study was approved by the Hospital Ethics Committee, and patients voluntarily participated in the study and signed the informed consent

#### 2.2.2. Exclusion Criteria

1. The patients had mental disorders and could not cooperate with the study.
2. The patients died during first aid
3. The patients had congenital heart disease

### 2.3. Methods

Both groups underwent routine examination after admission, and the patients diagnosed with AMI received anticoagulant and antithrombotic drugs.

Group Q was treated with meglumine adenosine cyclophosphate (manufacturer: Yabao Pharmaceutical Group Co., Ltd.; NMPA approval No.: H20058049; specification: 180 mg). 180 mg of meglumine adenosine cyclophosphate was mixed with 200 ml of 5% glucose injection for intravenous drip, once a day. The patients received continuous treatment for 7 days to observe the effect [19–21].

Group J was treated with meglumine adenosine cyclophosphate combined with ulinastatin (manufacturer: Guangdong Techpool Bio-Pharma Co., Ltd.; NMPA approval No.: H19990133). 100,000 IU of ulinastatin injection was mixed with 500 ml of 5% glucose solution for intravenous drip, once a day. The patients received continuous treatment for 7 days to observe the curative effect.

### 2.4. Observation Indexes

The treatment efficiency, cardiac structure indexes, cardiac systolic function, blood lipid levels, vascular endothelial function, QLI (quality of life) scores, BI indexes, and FMA (motor function) scores were compared.

The patients' condition was initially controlled with no adverse reactions during treatment, and all indexes gradually returned to normal after treatment, which was markedly effective. The patients had no obvious adverse reactions during treatment, and the indexes gradually returned to normal as expected, which was effective. The patients had serious adverse reactions, and the results of electrocardiogram and ultrasonic testing showed the risk of morbidity in the indexes, which was ineffective.

The cardiac systolic function included left ventricular ejection fraction (LVEF) and left ventricular fractional shortening (LVFS). Blood lipid included triglyceride (TG), total cholesterol (TC), low-density lipoprotein (LDL), and high-density lipoprotein (HDL). The vascular endothelial function was mainly to detect the content of PGI2, NO, and tPA. PGI2 could relax blood vessels, NO could relax blood vessels with anticoagulation function, and tPA could dissolve thrombus to some extent.

With a total score of 100 points, FMA motor function score can detect the upper limb function (66 points) and lower limb function (34 points). A higher score represented better motor function. The total score of the BI index was 100 points. A score of 100 points showed that patients could take care of themselves independently. 61-99 points showed that patients needed occasional care from others and could basically take care of themselves. 41-60 points showed that patients needed care from others in most cases and could hardly take care of themselves, and a score below 40 points showed that patients could not take care of themselves at all and needed intensive care. QLI (quality of life) scoring criteria included daily activities, work and life, and interpersonal relationships. Each criterion had a full score of 10 points, and a higher score represented the better quality of life.

### 2.5. Statistical Processing

In this study, the data was processed by SPSS20.0 and graphed by GraphPad Prism 7 (GraphPad Software, San Diego, USA). The dataset included enumeration data and measurement data. The measurement data were expressed as $\bar{x}\pm s$, tested by *t* test while the enumeration data were expressed as [*n*(%)], tested by *χ*^2^. The difference was statistically significant when *P* < 0.05.

## 3. Results

### 3.1. Comparison of Treatment Efficiency

Comparison of treatment efficiency showed that the treatment efficiency in group J was notably higher compared with group Q, with statistical significance (*P* < 0.05), as below.  Figure 1(a) shows the treatment efficiency of group J, in which 40 cases were markedly effective, 9 cases were effective, and 1 case was ineffective. The total treatment efficiency was 98%.  Figure 1(b) shows the treatment efficiency of group Q, in which 26 cases were markedly effective, 11 cases were effective, and 13 cases were ineffective. The total treatment efficiency was 74%.

### 3.2. Comparison of Cardiac Structure Indexes

Comparison of cardiac structure indexes showed that AD, IVS, LVIDs, and PWTs in group J were notably lower compared with group Q, with statistical significance (*P* < 0.05), as shown in Figure 2.

### 3.3. Comparison of Cardiac Systolic Function

Comparison of cardiac systolic function showed that LVFS and LVEF in group J were notably higher compared with group Q, with statistical significance (*P* < 0.05), as shown in Figure 3.

### 3.4. Comparison of Blood Lipid Levels

Comparison of blood lipid levels showed that TG, TC, LDL, and HDL in group J after treatment were notably lower compared with group Q, with statistical significance (*P* < 0.05), as shown in Table 2.

### 3.5. Comparison of Vascular Endothelial Function

Comparison of vascular endothelial function showed that the vascular endothelial function in group J was notably better compared with group Q, with statistical significance (*P* < 0.05), as shown in Table 3.

### 3.6. Comparison of QLI Scores, BI Indexes, and FMA Scores

Comparison of QLI scores, BI indexes, and FMA scores showed that the QLI score, BI index, and FMA score in group J were notably higher compared with group Q, with statistical significance (*P* < 0.05), as shown in Figure 4.

## 4. Discussion

After the onset of AMI, patients often suffer from obvious manifestations such as angina pectoris, palpitations, and dyspnea. In case of such manifestations, patients should go to the hospital for diagnosis and treatment immediately. After admission, AMI patients will be examined and diagnosed in the hospital according to their specific condition. The patients will be mainly examined by electrocardiogram, ultrasonic diagnosis, and CT diagnosis to determine whether the patients suffer from AMI [22–24]. To further explore the effect of their combination on cardiac function and endothelial function of AMI patients, in this paper, AMI patients were chosen as the research objects and treated with meglumine adenosine cyclophosphate only and meglumine adenosine cyclophosphate combined with ulinastatin. The treatment efficiency, cardiac structure indexes, cardiac systolic function, blood lipid levels, vascular endothelial function, QLI scores, BI indexes, and FMA scores were compared.

This study showed that the treatment efficiency, QLI score, BI index, and FMA score in group J were notably higher compared with group Q (*P* < 0.05). With the greatly reduced quality of life and living ability after the onset of AMI, patients can only stay in bed during treatment and even cannot complete the basic movements, and their limb motor function and limb flexibility will be affected to a certain extent. Evaluating quality of life, living ability and limb function in patients can timely obtain the changes of their physical condition from onset to treatment, thus indirectly confirming the therapeutic effect. The above results revealed that the treatment efficiency, quality of life, BI index, and limb function of patients treated with ulinastatin combined with meglumine adenosine cyclophosphate were notably improved.

The cardiac structure indexes, cardiac systolic function, blood lipid level, and vascular endothelial function in group J were notably better compared with group Q (*P* < 0.05). Cardiac structure indexes, cardiac systolic function, and vascular endothelial function can determine the changes of heart in AMI patients after the onset. Some patients with more serious conditions may show great changes in cardiac structure and atrioventricular diameter, which is unfavorable to the maintenance of vital movement. The heart works through constant contraction and relaxation, in which the heart pumps blood to all parts of the body during contraction, and blood flows back to the heart during relaxation to complete the blood circulation. Since hyperlipidaemia can also lead to cardiovascular and cerebrovascular diseases, timely monitoring and controlling blood lipid levels can prevent and control the related diseases. In the study of Song et al. [16], AMI patients were divided into group A treated with meglumine adenosine cyclophosphate and group B treated with ulinastatin combined with meglumine adenosine cyclophosphate. Their results showed that the number of angina attacks, duration of each attack, and cardiac function indexes in group B were notably better compared with group A, with a higher effective rate in group B. Their results are consistent with this study and fully proves the scientific and reliable results of this study.

## 5. Conclusion

In conclusion, ulinastatin combined with meglumine adenosine cyclophosphate can obviously enhance the therapeutic effect of AMI patients and improve the endothelial function and cardiac function, which should be widely applied in the clinic. However, there are still several shortcomings in our study. We need to collect more data and conduct deeper experiments to improve the analysis accuracy.

## Figures and Tables

**Figure 1:** Comparison of treatment efficiency Note: ∗ indicated the comparison of treatment efficiency between group J and group Q, with statistical significance (*χ*^2^ = 11.96, *P* < 0.001).

**Figure 2:** Comparison of cardiac structure indexes. Note: The abscissa from left to right represented AD, IVS, LVIDs, and PWTs, and the ordinate represented the measured data (mm). ∗ represented the comparison of AD between group J (15.93 ± 1.11) mm and group Q (17.00 ± 1.15) mm, with statistical significance (*t* = 4.73, *P* < 0.001). ∗∗ represented the comparison of IVS between group J (9.28 ± 0.66) mm and group Q (10.51 ± 0.79) mm, with statistical significance (*t* = 8.45, *P* < 0.001). ∗∗∗ represented the comparison of LVIDs between group J (39.66 ± 3.57) mm and group Q (43.87 ± 3.9) mm, with statistical significance (*t* = 5.63, *P* < 0.001). ∗∗∗∗ represented the comparison of PWTs between group J (10.02 ± 0.81) mm and group Q (11.74 ± 1.00) mm, with statistical significance (*t* = 9.45, *P* < 0.001).

**Figure 3:** Comparison of cardiac systolic function. Note: The abscissa from left to right represented LVFS and LVEF, and the ordinate represented the measured data (%). ∗ represented the comparison of LVFS between group J (35.20 ± 4.34) % and group Q (31.19 ± 4.28) %, with statistical significance (*t* = 4.65, *P* < 0.01). ∗∗ represented the comparison of LVEF between group J (52.29 ± 5.97) % and group Q (48.04 ± 5.31) %, with statistical significance (*t* = 3.76, *P* < 0.001).

**Figure 4:** Comparison of QLI scores, BI indexes, and FMA scores. Note: The abscissa from left to right represented FMA, QLI, and BI, and the ordinate represented the score (points). ∗ represented the comparison of FMA scores between group J (60.80 ± 4.25) and group Q (54.69 ± 4.97), with statistical significance (*t* = 6.60, *P* < 0.001). ∗∗ represented the comparison of QLI scores between group J (66.27 ± 8.80) and group Q (60.59 ± 8.22), with statistical significance (*t* = 3.34, *P* < 0.01). ∗∗∗ represented the comparison of BI scores between group J (72.04 ± 8.43) and group Q (67.49 ± 8.48), with statistical significance (*t* = 2.69, *P* = 0.008).

**Table 1:** Comparison of general data $\left(\bar{x}\pm s\right)$.

Items	Group J	Group Q	*χ* ^2^/*t*	*P*
Gender (male/female)	26/24	27/23	0.04	0.84
Age (years old)	62.34 ± 3.42	62.61 ± 3.58	0.39	0.70
Height (cm)	165.33 ± 10.32	164.87 ± 10.21	0.22	0.82
Weight (kg)	69.90 ± 8.84	69.85 ± 8.22	0.03	0.98
Heart disease history (years)	5.33 ± 1.06	5.19 ± 1.12	0.64	0.52
Time from onset to treatment (h)	1.30 ± 0.26	1.35 ± 0.33	0.84	0.40
Hypertension (*n*)	19	18	0.04	0.84
Hyperlipemia (*n*)	16	14	0.19	0.66

**Table 2:** Comparison of blood lipid levels $\left(\bar{x}\pm s,\text{mmol}/\text{L}\right)$.

Group	TG	TC	LDL	HDL
Group J	3.42 ± 0.59	0.94 ± 0.08	1.55 ± 0.30	1.19 ± 0.10
Group Q	5.31 ± 1.17	1.18 ± 0.14	2.31 ± 0.39	1.52 ± 0.23
*t*	10.20	10.52	10.92	9.30
*P*	<0.001	<0.001	<0.001	<0.001

**Table 3:** Comparison of vascular endothelial function $\left(\bar{x}\pm s\right)$.

Group	PGI2 (*μ*mol/L)	NO (pg/L)	tPA (ng/L)
Group J	65.33 ± 9.90	26.07 ± 5.81	20.08 ± 1.39
Group Q	57.48 ± 8.85	23.02 ± 5.24	17.14 ± 1.15
*t*	4.18	2.76	11.52
*P*	<0.001	0.007	<0.001

## Data Availability

The datasets used and/or analyzed during the current study are available from the corresponding author on reasonable request.
